# Comparison of Different Furosemide Regimens in the Treatment of Acute Heart Failure: A Meta-Analysis

**DOI:** 10.1155/2022/4627826

**Published:** 2022-08-18

**Authors:** Youpan Huang, Feijie Guo, Daori Chen, Haiman Lin, Jian Huang

**Affiliations:** ^1^Department of Emergency, People's Hospital of Wanning, Hainan, Wanning 571500, China; ^2^Department of Cardiovascular Medicine, Lingshui Li Autonomous County People's Hospital, Lingshui 572400, China; ^3^Department of Critical Care Medicine, People's Hospital of Wanning, Hainan, Wanning 571500, China

## Abstract

**Background:**

To compare the effects of different dosing schemes of furosemide on acute heart failure (AHF).

**Methods:**

Literature that compared the efficacy of continuous and intermittent administration of furosemide in AHF patients was retrieved from PubMed, Embase, the Cochrane Library, and ISI Web of Science from inception to May 2022. The primary endpoints included overall weight loss, 24-hour urine volume, length of hospital stay, 24-hour brain natriuretic peptide (BNP) level change, and all-cause mortality. The RevmMan5.4 software was used to analyze the extracted data.

**Results:**

A total of 10 studies with 775 patients, including 338 receiving continuous furosemide administration and 387 receiving intermittent furosemide administration, were included. The analysis results showed significant differences in weight loss (MD = 1.08, 95% CI (0.75~1.40), *P* < 0.00001) and 24-hour urine volume (MD =335.23, 95% CI (140.98~529.47), *P* = 0.0007) between the 2 groups. There was no significant difference in terms of length of hospital stay (MD = −0.71, 95% CI (-2.74~1.31), *P* = 0.49) and all-cause mortality (RR = 1.59, 95% CI (0.92~2.75), *P* = 0.10).

**Conclusions:**

Compared with intermittent administration, continuous infusion of furosemide had a significant effect on the 24-hour urine volume and total weight loss in patients with AHF.

## 1. Introduction

Acute heart failure (AHF) is a life-threatening clinical syndrome characterized by rapid deterioration of heart function caused by structural and/or functional cardiac abnormality that is associated with significant morbidity and mortality. The prevalence of heart failure varies with a specific region and population. In developed countries, the prevalence of AHF varies from 1.5% to 2.0% for the general population, and the incidence in people aged over 70 is even higher than 10% [1]. Studies have shown that AHF represents an enormous economic burden to both the families and society in terms of emergency admission, readmission, and prolongation of hospital stay [2].

Fluid retention is a typical consequence of heart failure caused by impaired cardiac contraction. In the current clinical practice, intravenous diuretics are fundamental for the treatment of AHF, with about 90% of hospitalized AHF patients receiving diuretics to reduce fluid retention and improve oxygenation [3, 4]. However, available data on the use of intravenous diuretics are predominantly limited to expert opinions and prospective studies that investigated that the optimal administration mode and dosage remain controversial. Studies have shown that large doses of diuretics were associated with adverse effects, such as activation of the angiotensin system and sympathetic nervous system, electrolyte disorder, and deterioration of renal function [5]. Associations between high-dose diuretics and adverse clinical outcomes, including renal failure, heart failure deterioration, and death, were noted [5]. In addition, the optimal mode of administration has always been controversial. Data suggested that continuous infusion has potential benefits such as decongestion compared with intermittent injection [6, 7]. Although some studies have evaluated the role of continuous infusion of diuretics for patients with heart failure [7–9], there have been some studies supporting that circulatory continuous infusion of diuretics can better help patients with diuresis; these studies have not reached consistent conclusions due to differences in sample size, infusion duration, and dose, and there are still some controversies. Therefore, in this paper, we conducted a meta-analysis of multiple literatures. Therefore, we conducted this systematic review and meta-analysis to compare the differences in total weight loss, 24-hour urine volume, length of hospital stay, and mortality between continuous intravenous furosemide infusion and intermittent injection.

## 2. Materials and Methods

### 2.1. Literature Search

Databases such as PubMed, Embase, the Cochrane Library, and ISI Web of Science were searched from the inception to May 2022. Studies that compared the effects of different dosing schemes of furosemide for AHF were collected. The search terms were “Acute heart failure”, “AMF”, “diuretics”, “Furosemide”, “Loop diuretics”, and “Continuous infusion”. The joint search was conducted with Medical Subject Headings (MESH) and free words. References to the target literature were also examined.

### 2.2. Inclusion and Exclusion Criteria

Inclusion criteria were as follows: (1) study type: randomized controlled trials (RCTs); (2) participants: hospitalized AHF patients, regardless of race, nationality, and gender; (3) intervention group: furosemide continuous infusion; (4) control group: intermittent injection of furosemide every 12 hours; and (5) outcomes: the primary endpoints were the overall weight loss, 24-hour urine volume, length of hospital stay, 24-hour brain natriuretic peptide (BNP) level changes, and all-cause mortality. Exclusion criteria were as follows: (1) non-RCT or animal studies, (2) studies with patient overlap, (3) literature with incomplete data or no indicators, and (4) subjects receiving diuretics other than furosemide.

### 2.3. Data Extraction and Quality Control

Potentially eligible RCTs were independently screened and cross-checked by Huang and Guo. Disagreements were resolved through discussion or consultation with Huang. Data extraction included the following: (1) general information: title, first author, publication time, and country; (2) patient demographics, clinical characteristics, laboratory test results, physical examination indicators, previous personal history, medical history, treatment history, and interventions of subjects; (3) risk of bias assessment indicators, including method of randomization, blinding of assignment and outcome assessment, completeness of outcome data, and selective reporting; and (4) outcomes of interest, including overall weight loss, 24-hour urine output, length of hospital stay, and 24-hour BNP.

RevMan 5.4 software was used to evaluate the quality of RCTs included. The risk of bias assessment table included the following items: random allocation method, allocation concealment scheme, blind method, blind method of result evaluation, the integrity of result data, selective report, and other biases.

### 2.4. Statistical Methods

RevMan 5.4 software was used for meta-analysis. Two-sided *P* < 0.05 indicated statistical significance. The mean difference (MD) and relative risk ratio (RR) with 95% confidence interval (CI) were used to analyze the continuous variables and binary variables, respectively. The *I*^2^ was used to test the interstudy heterogeneity. In the presence of no obvious heterogeneity (*P* > 0.05 and *I*^2^ < 50%), the fixed effects model was applied. Otherwise, the random effects model was used to explore the source of heterogeneity with subgroup analysis. Egger's test was used to evaluate the publication bias.

## 3. Results

### 3.1. Literature Search Results

A total of 1628 English publications were obtained through database retrieval. After screening and eliminating duplicate literature, 823 were obtained. The title and abstract of the literature were read, and articles that did not meet the inclusion/exclusion criteria were excluded. The remaining 86 publications were downloaded for full-text reading. Finally, 10 studies were included. The study flow chart is shown in Figure 1.

### 3.2. Study Subject Demographics

The included 10 studies compared the continuous intravenous injection of furosemide with furosemide intermittent injection in hospitalized AHF patients [8–17]. Studies were performed in Asia, Europe, North America, and Africa, with 3 from the United States [10–12], 2 from Italy [8, 9], and 1 from China [13], Turkey [14], India [15], Israel [16], and Egypt [17], respectively. The largest sample, with a total of 308 cases, was reported from the United States [11] (Table 1). A total of 775 patients were included, with 388 in the intervention group and 387 in the control group.

### 3.3. Weight Loss

A total of 7 studies [8–14] with 655 AHF patients reported overall weight loss during hospitalization. The fixed effects model was used for analysis, given the absence of interstudy heterogeneity (*I*^2^ = 0%, *P* = 0.90, Figure 2). The results showed that compared with intermittent administration, continuous injection of furosemide was associated with significantly more pronounced overall weight (kg) loss in AHF patients during hospitalization (MD = 1.08, 95% CI (0.75~1.40), *P* < 0.00001) (Figure 2). Egger's test showed no publication bias among the literature (*P* > 0.05).

### 3.4. Length of Hospital Stay

Seven studies [9–15] included 657 AHF patients and reported the length of hospital stay. The result of the heterogeneity test was *P* < 0.00001 and *I*^2^ = 84% (Figure 3). There was significant heterogeneity among the studies, which was analyzed by the random effects model. The results showed that compared with intermittent administration, there was no difference in hospital stay (days) between continuous administration and AHF patients (MD = −0.71, 95% CI (-2.74~1.31), *P* = 0.49) (Figure 3). Egger's test showed no publication bias among the literature (*P* > 0.05).

### 3.5. 24-Hour Urine Volume

24-hour urine volume was reported in 216 AHF patients from 4 studies [8, 9, 12, 16]. In the absence of significant heterogeneity (*I*^2^ = 19%, *P* = 0.30, Figure 4), the fixed effects model was used. Compared with intermittent administration, continuous administration was associated with significantly increased 24-hour urine volume (mL) in AHF patients (MD =335.23, 95% CI (140.98~529.47) (Figure 4). No publication bias was noted (*P* > 0.05).

### 3.6. 72-Hour Urine Volume

In total, 3 studies [10, 11, 13] with 230 AHF patients reported 72-hour urine volume. There was significant heterogeneity among the studies (*I*^2^ = 89%, *P* = 0.0002, Figure 5), which were analyzed by the random effects model. There was no significant difference in 72-hour urine volume (mL) between the continuous administration group and the intermittent injection group (MD =494.29, 95% CI (-671.43.05~1660.00), *P* = 0.41) (Figure 5). Egger's test showed no publication bias among the literature (*P* > 0.05).

### 3.7. Changes in BNP Level

Meta-analysis of 221 AHF patients from 3 studies [8, 9, 13] using the random effects model (*I*^2^ = 71%, *P* = 0.03, Figure 6) showed that continuous administration of furosemide was not associated with significantly decreased BNP levels (pg/mL) as compared with the furosemide intermittent injection (MD = 86.97, 95% CI (-117.31~291.24), *P* = 0.40) (Figure 6). Egger's test showed no publication bias among the literature (*P* > 0.05).

### 3.8. All-Cause Mortality

All-cause mortality was reported in 531 AHF patients from 5 studies [9, 11, 12, 15, 17] without obvious interstudy heterogeneity (*I*^2^ = 0%, *P* = 0.59, Figure 7). No significant differences in terms of all-cause mortality were observed between continuous administration and intermittent administration (RR = 1.59, 95% CI (0.92~2.75), *P* = 0.10) (Figure 7). Egger's test showed no publication bias among the literature (*P* > 0.05).

## 4. Discussion

AHF is a multietiological clinical syndrome characterized by sudden decrease in heart function. People over 70 years old have a higher incidence that can reach over 10%, causing substantial economic costs to the families and society [1, 2]. Currently, intravenous diuretics are still the primary treatment for AHF. Nonetheless, the optimal dosing regimen has not been determined.

In this meta-analysis, we found that compared with intermittent administration, continuous injection of furosemide could significantly reduce the weight of AHF patients. In addition, the 24-hour urine volume increased more significantly in hospitalized AHF patients receiving continuous furosemide administration. No significant differences were found in terms of the length of hospital stay, BNP level, and all-cause mortality between the two groups.

Our study showed that continuous administration can increase patients' urine volume, which is consistent with the results of previous analyses by Amer et al. [18], Kuriyama et al. [19], and Ng et al. [20]. In addition, there was no obvious heterogeneity in the studies. Among all the observation indicators, the data on patients' weight change during hospitalization in each study was the most complete, which might be related to the convenience of weight measurement. Therefore, continuous injection of furosemide can reduce patients' weight better than intermittent injection of furosemide.

In treating AHF, increasing the urine output is an important treatment goal. Our study showed that continuous administration can significantly increase the 24-hour urine volume but not the 72-hour urine volume. However, it should be noted that only three studies with significant interstudy heterogeneity have reported 72-hour urine volume. Our study finding is consistent with the results of Amer [18] and Ng et al. [20], which also noted that continuous furosemide administration can reduce patients' weight during hospitalization. Theoretically [21], continuous administration maintains a stable furosemide concentration and exerts a continuous diuretic effect by targeting the renal tubules. In comparison, with intermittent administration, the effective level could be maintained for a limited time after drug injection, and most diuretics will be excreted within 2 h. Intermittent injection of a large dose of furosemide leads to rapid decline of blood volume, thus increasing the incidence of adverse reactions such as hypokalemia and hypotension [22].

BNP is predominantly synthesized and secreted by the left ventricular cardiomyocytes. Since BNP secretion is positively correlated with the severity of AHF, it is often used as an important biomarker and prognosticator of heart failure [23]. Therefore, we investigated the changes in BNP levels in AHF patients after continuous or intermittent furosemide administration. We found no significant difference between the two groups regarding BNP changes, which is consistent with the findings that the two administration methods showed no differences in length of hospital stay and the prognosis of AHF. Additional studies with larger sample are needed to compare the 2 dosing regimens in terms of BNP level changes, hospital stay, and all-cause mortality.

Although continuous furosemide administration can promote the elimination of excessive body fluids and reduce body weight more efficiently, it did not improve the prognosis of AHF. Theoretically [24], continuous infusion of furosemide should be more conducive to weight loss and urine output and accelerate the reduction of cardiac congestive symptoms. AHF is a multifactorial disorder that cannot be prognosticated solely by eliminating body fluid volume. The use of furosemide can promote the elimination of body fluids and promote the excretion and loss of sodium, chlorine, potassium, calcium, magnesium, and phosphorus. Large dose of furosemide may cause water electrolyte disequilibrium, positional hypotension, shock, and related adverse reactions such as thirst, fatigue, muscle soreness, and arrhythmia [25], all of which may affect the prognosis of AHF. However, most studies did not include the changes in electrolytes as an observation indicator. Kuriyama et al. [19] found no significant difference between continuous and intermittent furosemide administration in terms of electrolyte changes in AHF patients through analysis of a few studies. Therefore, we believe that the change in electrolytes should also be studied as an important index of furosemide efficacy in AHF treatment.

The main advantages of this analysis lie in its precise definition, comprehensive retrieval strategy, and large sample size. Our limitation is that some results were heterogeneous, and some studies were not blind. The heterogeneity of the results was predominantly related to small sample size and different observation indicators among studies. In addition, the inclusion criteria also vary among studies. In the continuous injection group, furosemide was continuously injected by the intravenous pump. For intermittent administration, furosemide was taken orally whereas in others, it was injected intravenously. Due to the limited number of studies, we could only divide them into two groups based on whether it was continuous or intermittent administration. In addition, the specific dose of furosemide used in the treatment of AHF varies among studies, which might also be an important source of heterogeneity. Therefore, the benefits of continuous injection of furosemide need further experimental research and exploration. In conclusion, compared with intermittent injection, continuous intravenous injection of furosemide could promote excretion of excessive body fluid more effectively in AHF patients. However, there were no significant differences between the two groups with regard to length of hospital stay and mortality. The dosing regimen of furosemide in the treatment of AHF needs to be further explored.

## Figures and Tables

**Figure 1:** Document screening flow chart.

**Figure 2:** Forest chart of total weight loss between continuous intravenous injection and intermittent injection of furosemide.

**Figure 3:** Comparison forest chart of hospitalization days between continuous intravenous injection and intermittent injection.

**Figure 4:** Comparison forest chart of 24-hour urine volume between continuous intravenous injection and intermittent injection.

**Figure 5:** Comparison forest chart of 72-hour urine volume between continuous intravenous injection and intermittent injection.

**Figure 6:** Forest chart of BNP changes in patients with continuous intravenous injection and intermittent injection.

**Figure 7:** Forest chart of all-cause mortality in patients with continuous intravenous injection and intermittent intravenous injection.

**Table 1:** Basic information of included literature and risk of bias assessment.

Study/year	Country	Sample size	Design	Dose of daily furosemide (mg)	Duration of interventions (hours)	Outcomes used in meta-analysis	Risk of basis
Makhoul/1997 [16]	Israel	20	Single-centre RCT	cIV: 329 ± 186.7 iIV: 324 ± 110.8 (divided in 3 doses)	24	Total urine output in 24 h	Low risk

Allen/2010 [10]	USA	41	Single-centre RCT	cIV: 162 ± 48 iIV: 162 ± 52 (divided in 2 doses)	48	Changes in weight loss Length of hospital stay Total urine output in 72 h	Uncertain risk

Thomson/2010 [12]	USA	56	Single-centre RCT	cIV: 197 ± 148 iIV: 172 ± 97	100	Changes in weight loss	Uncertain risk
						Length of hospital stay	
						Total urine output in 24 h	
						Mortality	

Felker/2011 [11]	USA+Canada	308	Single-centre RCT	cIV: 162 ± 48 iIV: 162 ± 52 (divided in 2 doses)	72	Changes in weight loss Length of hospital stay Total urine output in 72 h Mortality	Uncertain risk

Shah/2014 [15]	India	60	Single-centre RCT	cIV: 100 iIV: 100 (divided in 2 doses)	48	Length of hospital stay Mortality	High risk

Yayla/2015 [14]	Turkey	29	Single-centre RCT	cIV: 160 iIV: 160 (divided in 2 doses)	48	Changes in weight loss Length of hospital stay	Uncertain risk

Palazzuoli/2014 [9]	Italy	82	Single-centre RCT	cIV: 170 ± 70 iIV: 160 ± 80	112	Changes in weight loss Length of hospital stay Total urine output in 24 h Changes in BNP Mortality	Uncertain risk

Palazzuoli/2015 [8]	Italy	58	Single-centre RCT	cIV: 165 ± 85 iIV: 165 ± 85 (divided in 2 doses)	120	Changes in weight loss Total urine output in 24 h Changes in BNP	Low risk

Ragab/2018 [17]	Egypt	40	Single-centre RCT	cIV: 120/240 iIV: 120/240 (divided in 3 doses)	24	Mortality	Uncertain risk

Zheng/2021 [13]	China	81	Single-centre RCT	cIV: 160/200 iIV: 160/200	72	Changes in weight loss Length of hospital stay Total urine output in 72 h Changes in BNP	Uncertain risk

Note: cIV: continuous intravenous; iIV: intermittent intravenous.

## Data Availability

The data used to support the findings of this study are included within the article.
